RETRACTED

# Mental Health Effects of Entrepreneurial College Students from Different Backgrounds: The Mediating Role of Social Equity

**DOI:** 10.1155/2022/4790284

**Published:** 2022-03-08

**Authors:** Dehui He, Wangzhuo Li, Xinghui He

**Affiliations:** ^1^Changde Vocational Technical College, Changde, China; ^2^Graduate School of Guangzhou University of Chinese Medicine, Guangzhou, China; ^3^Hunan Education Department, Changsha, China

## Abstract

In this study, the impact of entrepreneurial college students from different backgrounds on mental health which is primarily based on the mediating role of social justice is studied. For this purpose, we have selected those start-up students who graduated from a university for one to two years as the research object, and 1890 questionnaires were distributed. The subjective family background, objective family background, social equity perception, anxiety, and depression of entrepreneurial college students were investigated, and the results were analyzed. The level of social equity and mental health of start-up college students with better birth was significantly higher than that of start-up college students with lower birth. Background, social equity, and positive emotions were significantly positively correlated, which was significantly negatively correlated with negative emotions, depression, and anxiety; Social equity played a partial mediating role in the relationship between birth and mental health indicators. Social equity helped to maintain the mental health of entrepreneurial college students from different backgrounds. This was of great significance to the entrepreneurial college students who come from a lower background.

## 1. Introduction

People's demand for fairness, justice, rule of law, and other aspects is constantly increasing; of course, the existence of some social unstable factors also causes people to have different degrees of anxiety and insecurity [1]. Social equity and justice are the main line of value in the modernization process. At present, there is some resistance to promote the realization of social equity and justice in the modernization process of China. The deep-rooted reasons are that the reform process lags behind the development process, economic development alone cannot meet the needs of a better life, and the modernization process has only a single participant [2]. For this reason, it is necessary to promote the organic combination of reform and development through governance modernization and achieve social fairness and justice more effectively in historical development, comprehensive development, and shared development [3]. Entrepreneurial college students, as the main force of innovative and entrepreneurial talents, need to have a high ability of innovation and entrepreneurship in order to play a certain role in the development of social innovation in China. The promotion mechanism of innovation and entrepreneurship education should be reasonably constructed to promote the development of innovation and entrepreneurship education in colleges and universities, so as to promote the long-term development of entrepreneurial students [4, 5]. According to the social equity theory, this belief leads people to believe that the society they live in is stable and orderly; the results can be predicted; they will be treated fairly and will not be the victims of unforeseen disasters and various injustices. This provides people with a sense of security and control [6]. Only in this way can people feel confident about the future, pursue long-term goals, and believe that they will eventually get what they deserve. Thus, just society beliefs can serve as a personal resource to reduce the reverberations of injustice. Belief in social equity is particularly important for disadvantaged groups. Studies have found that belief in social equity has a greater impact on the emotions and life adaptation of entrepreneurial college students from different backgrounds [7]. A just society is of particular significance to low-background entrepreneurs because compared with high-level entrepreneurs, low-background entrepreneurs are more likely to be victims of various injustices. When investing in the future, they will consider equity, which means whether individuals have the opportunity to make a difference through their own efforts [8, 9]. Entrepreneurial college students are in an important stage of pursuing their life goals. Therefore, this study selected entrepreneurial college students as the research object and examined the influence of subjective and objective family background on the mental health of entrepreneurial college students. This study explored the role of social equity belief in the relationship between entrepreneurial college students from different backgrounds and mental health.

RETRACTED

In this study, the impact of entrepreneurial college students from different backgrounds on mental health which is primarily based on the mediating role of social justice is studied. For this purpose, we have selected those start-up students who graduated from a university for one to two years as the research object, and 1890 questionnaires were distributed. The subjective family background, objective family background, social equity perception, anxiety, and depression of entrepreneurial college students were investigated, and the results were analyzed. The level of social equity and mental health of start-up college students with better birth was significantly higher than that of start-up college students with lower birth. Background, social equity, and positive emotions were significantly positively correlated, which was significantly negatively correlated with negative emotions, depression, and anxiety. Social equity played a partial mediating role in the relationship between birth and mental health indicators.

The rest of the manuscript's sections are arranged according to the following plan which is provided in the following paragraph.

In subsequent section, i.e., Section 2, the proposed evaluation methods used to measure or judge the effectiveness of the student's mental health status and its impact on the entrepreneurial are provided. In Section 3, an experiment evaluation study is carried out and their results are reported which is followed by the brief discussion section. Finally, concluding remarks are given along with group of relevant references which are used in this manuscript.

## 2. Proposed Evaluation Method of the College Students

### 2.1. General Information

The entrepreneurial students who graduated from universities for one to two years were selected as the research objects.

### 2.2. Implementation Methodology

1890 questionnaires were sent out, and 1738 questionnaires were collected with a recovery rate of 91.96%. 12 discarded questionnaires were eliminated, and 1726 valid questionnaires were collected. Among them, 1226 were male (71.03%) and 500 were female (28.97%). They were between 19 and 25 years old.

### 2.3. Observational Index

To investigate the subjective family background, objective family background, social equity perception, anxiety, and depression of entrepreneurial college students.

#### 2.3.1. Subjective Family Origin Measurement

With reference to relevant studies [10], using a single measure, the question was as follows: where do you think your family is in society at the moment of birth? Participants were asked to rate their family background on a given set of five options: lower, lower middle, middle, upper middle, and upper middle. They were assigned a score of 1–5, and the higher the score was, the higher the class of family they believed they belonged to.

#### 2.3.2. Objective Measures of Family Origin

Five indicators were collected for this study:

- Annual household income (“5000 and below,” “5001–15000,” “15001–30000,” “30001–60000,” “60001–100000,” and “100000 and more” assign 1–6 points, respectively).
- Education level of mother and father (“Primary school or below,” “Junior high school (including not graduated),” “High school or technical secondary school (including not graduated),” “Junior college,” “Undergraduate,” and “Postgraduate (Master or Doctor);” they were assigned 1–6 points.
- The occupation of the mother and father (the ten origins based on the classification and the status of the occupation of organizational resources, economic resources, and cultural resources, assigned in turn to be 1–10 points).

RETRACTED

#### 2.3.3. Social Equity Scale

The self-subscale was used in this study and consisted of seven items, on a scale of 1–6 (1 = strongly disagree; 6 = strongly agree). In this study, the internal consistency coefficient of the subscale was 0.86.

#### 2.3.4. Self-Rating Anxiety Scale [11]

The 20 items were scored from 1 to 4. The standard score was used in this study. The higher the score, the more serious the anxiety.

#### 2.3.5. Self-Rating Depression Scale [12]

20 items were scored from 1 to 4, and the standard score was used in this study. The higher the score, the more severe the depression.

### 2.4. Statistical Methods

SPSS 21.0 statistical software was used. Measurement data were expressed as *x* ± *s*, and the *t* test was used. Enumeration data were expressed as frequency and percentage. The calibration test was conducted for enumeration data between groups with theoretical frequencies ≥0 and ≤5. The statistical data of theoretical frequency >5 between the groups were the *χ*^2^ test, and *P* < 0.05 indicated statistically significant difference.

## 3. Results and Evaluations

### 3.1. Comparison of Social Equity and Mental Health Status of College Students with Different Entrepreneurial Backgrounds

In order to compare whether there were differences in social equity and mental health of entrepreneurial college students from different backgrounds, the data were processed as follows: for the data of subjective family background, the subjects who self-reported their subjective family background as “lower class” were selected as the low subgroup and the subjects who self-reported their subjective family background as “upper class.” For objective family origin data, the subjects were first ranked according to their scores from highest to lowest; then, the *t*-test was carried out for high and low scores of subjective and objective family backgrounds, respectively. The results showed that, both subjectively and objectively, the social equity and mental health of entrepreneurial college students with higher family social background were significantly higher than those with lower family social background. Comparison of social equity and mental health status of college students with different entrepreneurial backgrounds is given in Table 1.

### 3.2. The Relationship between Family Background, Social Equity, and Mental Health of Entrepreneurial College Students

Subjective family background was significantly positively correlated with objective family background. Social equity was significantly positively correlated with both subjective and objective family background and was significantly positively correlated with life satisfaction and positive emotions. It was significantly negatively correlated with negative emotion, anxiety, and depression. At the same time, the subjective and objective family background and the above mental health indicators were also significantly positive correlation. The relationship between family background, social equity, and mental health of entrepreneurial college students is given in Table 2.

RETRACTED

### 3.3. Analysis of the Mediating Role of Social Equity

For family background, social equity, and negative emotional experience, the following fitting indexes were obtained by model fitting: *χ*^2^ = 10.962, DF = 3, *χ*^2^/DF = 3.645, GFI = 0.991, NFI = 0.993, IFI = 0.984, TLI = 0.994, CFI = 0.993, and RMSEA = 0.021. Among them, the path coefficient between family social background and negative emotional experience was significant, indicating that social equity plays a partial mediating role. The model showed that the direct effect of family social background on negative emotional experience was −0.092, the indirect effect mediated by social equity was −0.079, the total effect was −0.175, and the indirect effect accounted for 45.76% of the total effect. Normalized path diagram is shown in Figure 1.

## 4. Discussion

Forming a reasonable and orderly pattern of income distribution is an inevitable requirement for promoting social equity. In order to form a reasonable and orderly pattern of income distribution, on the one hand, it should continue to work for more and get more, focus on protecting income from work, increase the remuneration of workers, especially front-line workers, and increase the proportion of remuneration in primary distribution [13]. On the other hand, we will improve the mechanism whereby labor, capital, land, knowledge, technology, management, data, and other factors of production are assessed by the market, and remunerations are determined based on their contributions [14, 15]. The entrepreneurship of college students can help them realize successful entrepreneurship with the help of innovative ideas, contribute to the development of social economy, and realize their own life value [16]. Social equity plays a partial mediating role in the relationship between different birth backgrounds and mental health [17]. Family background reflects the differences in the resources occupied by the families of entrepreneurial students, which may directly lead to the disadvantage of entrepreneurial students in the future competition, thus generating psychological pressure [18, 19]. At the same time, this difference may also affect the mental health level of entrepreneurial college students through their perception of social equity [20]. The perception of social equity reflects the extent to which entrepreneurial students believe that they can change this disadvantage through their own efforts. If they believe that they can change the status quo of their birth through their efforts, they will experience less negative emotions, be full of confidence in the future, and be willing to pursue long-term goals [21, 22]. In establishing a family social class, the index of just society belief and mental health in the process of the structural equation found that while studying family social class, the subjective and the objective of the model fitting degree better, consistent with the existing results, shows that in exploring students' family social class's influence on its development, considering the main evaluation indicators may be more comprehensive and objective class. The results showed the following:

1. The level of social equity and mental health of start-up college students with better birth was significantly higher than that of start-up college students with lower birth
2. Family background and social equity were negatively correlated with negative emotion, depression, and anxiety
3. Social equity played a partial mediating role in the relationship between birth and mental health indicators

RETRACTED

## 5. Conclusion

In this study, the impact of entrepreneurial college students from different backgrounds on mental health which is primarily based on the mediating role of social justice is studied. For this purpose, we have selected those start-up students who graduated from a university for one to two years as the research object, and 1890 questionnaires were distributed. The subjective family background, objective family background, social equity perception, anxiety, and depression of entrepreneurial college students were investigated, and the results were analyzed. The level of social equity and mental health of start-up college students with better birth was significantly higher than that of start-up college students with lower birth. Background, social equity, and positive emotions were significantly positively correlated, which was significantly negatively correlated with negative emotions, depression, and anxiety. Social equity played a partial mediating role in the relationship between birth and mental health indicators. To sum up, social equity is helpful to maintain the mental health of entrepreneurial college students from different backgrounds, which is of great significance to entrepreneurial college students from lower backgrounds.

RETRACTED

## Figures and Tables

**Figure 1:** Normalized path diagram.

**Table 1:** Comparison of social equity and mental health status of college students with different entrepreneurial backgrounds.

Projects	Subjective family background			Objective family background		
	High score	Low score	*t*	High score	Low score	*t*
Perception of social equity	32.81	29.13	4.562	31.57	29.84	7.805
Anxiety	37.36	40.02	−5.831	37.02	39.31	−8.004
Depression	41.35	45.36	−7.240	42.11	44.57	−8.023

**Table 2:** The relationship between family background, social equity, and mental health of entrepreneurial college students.

Variable	M ± SD	Subjective family background	Objective family background	Perception of social equity	Anxiety	Depression
Subjective family background	2.42 ± 0.74	1.000				
Objective family background	0.00 ± 1.00	0.525	1.000			
Perception of social equity	30.75 ± 5.63	0.128	0.108	1.000		
Anxiety	38.33 ± 7.32	−0.083	−0.104	−0.372	1.000	
Depression	43.23 ± 9.20	−0.107	−0.111	−0.442	0.652	1.000

## Data Availability

The data used to support the findings of this study are included within the article.
